The article "Desensitization of TRPV1 Involved in the Antipruritic Effect of Osthole on Histamine-Induced Scratching Behavior in Mice" was published in 2021. Journal: Evid Based Complement Alternat Med.

# Desensitization of TRPV1 Involved in the Antipruritic Effect of Osthole on Histamine-Induced Scratching Behavior in Mice

**DOI:** 10.1155/2021/4012812

**Published:** 2021-10-13

**Authors:** Niuniu Yang, Ying Ju, Delun Huang, Kunhong Ling, Han Jin, Jiamin Liu, Jing Ma, Yongxin Chen, Yingge Zhang, Chan Zhu, Yan Yang, Zongxiang Tang, Xi Chen, Guanyi Wu

**Affiliations:** ^1^Department of Traditional Chinese and Western Medicine, College of Medicine, Yangzhou University, Yangzhou 225009, China; ^2^School of Medicine & Holistic Integrative Medicine, Nanjing University of Chinese Medicine, Nanjing 210023, China; ^3^College of Basic Medicine, Guangxi University of Chinese Medicine, Nanning 530299, China; ^4^College of Pharmacology, Guangxi Medical University, Nanning 530200, China

## Abstract

Osthole has been isolated from the fruits of *Cnidium monnieri* (L.) Cusson, which has been used in Chinese traditional medicine to treat pruritic disorders for a long time. However, the antipruritic mechanism of osthole is not fully understood. In the present study, using calcium imaging, molecular docking, and animal scratching behavior, we analyzed the pharmacological effects of osthole on transient receptor potential vanilloid 1 (TRPV1). The results showed that osthole significantly induced calcium influx in a dose-dependent manner in dorsal root ganglion (DRG) neurons. Osthole-induced calcium influx was inhibited by AMG9810, an antagonist of TRPV1. Osthole and the TRPV1 agonist capsaicin-induced calcium influx were desensitized by pretreatment with osthole. Furthermore, molecular docking results showed that osthole could bind to TRPV1 with a hydrogen bond by anchoring to the amino acid residue ARG557 in the binding pocket of TRPV1. In addition, TRPV1 is a downstream ion channel for the histamine H1 and H4 receptors to transmit itch signals. Osthole attenuated scratching behavior induced by histamine, HTMT (histamine H1 receptor agonist), and VUF8430 (histamine H4 receptor agonist) in mice. These results suggest that osthole inhibition of histamine-dependent itch may be due to the activation and subsequent desensitization of TRPV1 in DRG neurons.

## 1. Introduction

The transient receptor potential vanilloid member 1 (TRPV1) channel is a well-known subfamily the TRP ion channel family, comprising nonselective cation ion channels [1], expressed on a large subset of cutaneous and sensory neurons in the dorsal root ganglion (DRG) that responds to noxious stimulation. TRPV1 plays a role in mediating acute and chronic itch stimulated by histamine and other pruritogens, such as bradykinin, IL-31, and LTB4 [2, 3]. Injecting trypsin into TRPV1^−/−^ mice resulted in a significant reduction in scratching behavior [4]. Histamine activates H1R and H4R in DRG neurons via the PLC*β*/PKC pathway and/or the PLA2/lipoxygenase (LO) pathway and finally coupled to TRPV1 [5–7]. Previous studies have demonstrated that both antagonists and agonists of TRPV1 can lead to pain or itch relief through inactivation and chronic desensitization. Topically applied capsaicin (0.025%) can effectively treat moderate and severe pruritus induced by psoriasis [8, 9] and exert moderate restraint effects on itch responses induced by histamine, substance P, and PAR-2 agonist [10]. Furthermore, 8% topical capsaicin patches also have a therapeutic effect in chronic pruritus [11, 12], thus making targeting TRPV1 an attractive strategy for itch therapy.

*Cnidii monnieri* Fructus (dried fruit of *C. monnieri* (L.) Cusson), known as “She chuang zi” in China, was widely applied in the clinical practice of Traditional Chinese Medicine for treating diseases such as morbid leucorrhea, lumbago, vulva eczema, vulva itch, trichomonas vaginitis, impotence, cold uterus, and cold-dampness [13, 14]. It has been reported that the ethanol extract of *Cnidii monnieri* Fructus, including osthole (7-methoxy-8-isopentenoxycoumarin, Figure 1), showed an inhibitory effect on compound 48/80-induced scratching behavior [15]. Osthole is a major constituent of *Cnidii monnieri* Fructus, which plays a role in delaying the occurrence of Alzheimer's disease and has anti-inflammatory, antipruritic, antioxidant, antiallergic, anticancer, and antiosteoporotic effects [16–21]. Research has shown that osthole can alleviate diabetic neuropathic pain through the P2X4 receptor and suppress the expression of acid-sensing ion channel 3 (ASIC3) in rat DRG to alleviate nucleus pulposus-evoked nociceptive responses [22, 23]. Furthermore, osthole attenuates mouse atopic dermatitis by inhibiting thymic stromal lymphopoietin (TSLP) production in keratinocytes [19]. Our previous study showed that osthole could inhibit histamine-dependent itching by modulating TRPV1 [24]. However, osthole-activated TRPV1 in DRG neurons has not yet been clarified. TRPV1 is the downstream channel of itch signal transduction, and it is interesting how osthole exerts its antipruritic effect through TRPV1 activation. In addition, it is important to understand the antipruritic function of *C. monnieri* Fructus.

In this study, we found that osthole can activate TRPV1 in DRG neurons and is inhibited by AMG9810 (an antagonist of TRPV1). Furthermore, the scratching behavior induced by histamine, HTMT, and VUF8430 restrained by osthole may be due to desensitization of TRPV1.

## 2. Materials and Methods

### 2.1. Animals

A total of 60 male and female C57BL/6 mice aged 8 weeks were used for itch behavioral testing and calcium imaging. The animals were housed in a temperature-controlled room (22 ± 2°C) under a 12-hour light/dark cycle, with free access to food and water. All experiments were performed in accordance with the relevant guidelines and regulations approved by the Institutional Animal Care and Use Committee of Yangzhou University, Guangxi University of Chinese Medicine (Ethics license DW20181220-153), and Nanjing University of Chinese Medicine (Ethics license ACU190601, 20,190,605).

### 2.2. Culture of Dissociated DRG Neurons

After C57BL/6 mice were anesthetized with 4% isoflurane, acutely dissociated DRG neurons were collected in cold DH10 (90% Dulbecco's modified Eagle's medium (DMEM)/F-12, 10% fetal bovine serum (FBS), penicillin (100 U/ml), and streptomycin (100 *μ*g/ml), Gibco) and treated with an enzyme solution (dispase (5 mg/ml), collagenase type I (1 mg/ml) in Hanks' balanced salt solution (HBSS) without Ca^2+^ and Mg^2+^, Gibco) at 37°C for 30 min. After breakup and centrifugation, cells were resuspended in DH10, plated on glass coverslips coated with poly-D-lysine (0.5 mg/ml) and laminin (10 *μ*g/ml, Invitrogen), and cultured in an incubator (95% O_2_ and 5% CO_2_) at 37°C [25].

### 2.3. Calcium Imaging

Dorsal root ganglia were dissociated and cultured from mice for 16–18 h. For calcium imaging experiments, cells were loaded with fura-2-acetomethoxyl ester (Molecular Probes) in HBSS solution for 30 min in the dark at room temperature, 26°C [25]. After washing three times, cells were imaged at 340 nm and 380 nm excitation to detect intracellular free calcium. Normal solution: 140 mM NaCl, 5 mM KCl, 10 mM HEPES, 2 mM CaCl_2_, 2 mM MgCl_2_, 10 mM D-(+)-glucose, and pH 7.4 with NaOH. Baseline readings were taken at 20 s before applying osthole or capsaicin to DRG neurons.

### 2.4. Molecular Docking

Interaction between osthole and TRPV1 was analyzed in silico using molecular docking by AutoDock 4.2.6.

#### 2.4.1. Molecular and Protein Structure Preparation

The three-dimensional structure of the target TRPV1 protein was obtained from the Protein Data Bank (5IRZ) (PDB, https://www.rcsb.org/). The TRPV1 ligands phosphatidylinositol and osthole were used in the MOPAC program to optimize the molecular structure and calculate the AM1 atomic charge. All protein and molecular structures were prepared using AutoDock Tools 1.5.6, and the corresponding pdbqt file was generated for docking preparation.

#### 2.4.2. Molecular Docking Method

AutoDock 4.2.6 software was used to perform the molecular docking experiments [26]. First, the docking grid box sizes were 50 × 50 × 60 for TRPV1 with a default spacing of 0.375 Å, and the *x*, *y*, *z* center was (126.562 135.846 104.054). Second, the grid point energy of the docking area was calculated using the AutoGrid program. The Lamarckian genetic algorithm (LGA) method was employed for docking experiments. The number of GA runs was 100, the population size was 150, and the maximum number of iterations. The maximum number of evaluations was 25000000. All other parameter values were set to the default for AutoDock 4.2.6. All calculations were performed using the MolDesigner molecular simulation platform. All results were analyzed using PyMol. PoseView created a two-dimensional schematic representation [27]. The three-dimensional structure of the protein and ligand was created using PyMol. Chimera created a hydrophobic surface schematic representation.

### 2.5. Scratching Behavior Assays

To measure scratching behavior, the model was described by Kuraishi et al. [28]. Mice were randomized into two groups: the osthole group and the control group. The rostral and dorsal necks of mice were clipped and depilated with an electric hair clipper two days before the experiments. Mice were placed in a transparent plastic box (4.5 × 4.5 × 7 inches) for approximately 30 min to avoid acclimatization before each experiment. The animals in the osthole group were subcutaneously injected with 1 *μ*M osthole in a volume of 100 *μ*l, as the control group animals received 100 *μ*l of equivalent vehicle solution (DMSO, 1‰) without osthole. Histamine or histamine H1 receptor agonist HTMT and histamine H4 receptor agonist VUF 8430 were injected into the nape of the mouse neck 30 min later. One scratch response was defined as the lifting of the hind limb towards the injection site. In all experiments, videotapes were played back, and the number of scratch bouts was counted at 5 min intervals for 30 min by an investigator blinded to the treatments.

### 2.6. Drugs and Compounds

Osthole was obtained from Shanghai YuanYe Biotechnology Co., Ltd. (Shanghai, China). Histamine, histamine trifluoromethyl toluidide (HTMT), capsaicin, VUF 8430 dihydrobromide, and AMG9810 were obtained from Sigma-Aldrich Corp. (St. Louis, MO, USA). All drugs were dissolved in dimethyl sulfoxide (DMSO) or saline. The drugs were diluted in saline used in the scratching experiments or normal perfusion solution in the calcium imaging experiments. The final concentrations of DMSO or water did not exceed 0.5%.

### 2.7. Statistical Analysis

All data were expressed as mean ± S.E.M. Differences among the groups were evaluated by the *t*-test and one-way analysis of variance (ANOVA) with Dunnett's multiple comparison test. A result with *P* ≤ 0.05 was considered “significantly different.”

## 3. Results

### 3.1. Osthole Activated DRG Neurons in a Concentration-Dependent Manner

To investigate the effect of osthole on DRG neurons, calcium fluorescence imaging was performed to confirm the speculation and effect of osthole on DRG neurons in vitro as previously described [18]. The results showed that pretreatment of 30 *μ*M osthole three times can stimulate Ca^2+^ transients (0.34 ± 0.03 (first), 0.22 ± 0.05 (second), and 0.15 ± 0.05 (third) (^*∗∗*^*P* < 0.01, one-way ANOVA followed by Dunnett's test versus Ost 1st), fluorescence ratio 340 nm/380 nm) in the same DRG neurons repeatedly (9.50% positive cells in total cells, *n* = 3 animals), which suggests that the activation effect of osthole was reversible (Figure 2). Furthermore, 10 *μ*M (9.02% positive cells in total cells, *n* = 3 animals), 30 *μ*M (17.93% positive cells in total cells, *n* = 3 animals), and 100 *μ*M (29.28% positive cells in total cells, *n* = 3 animals) osthole dose-dependently stimulated Ca^2+^ influx (^*∗*^*P* < 0.05, *t*-test, 10 *μ*M osthole versus 30 *μ*M osthole; 30 *μ*M osthole versus 100 *μ*M osthole) (Figure 3). While perfusing with calcium-free extracellular fluid, DRG neurons cannot be activated by osthole at a dose of 30 *μ*M (*n* = 3 animals) (data not shown). This indicates that osthole can activate DRG neurons dependent on extracellular Ca^2+^ influx.

### 3.2. Osthole Bound to TRPV1 *In Silico*

In our previous study, we demonstrated that osthole inhibits histamine-dependent itch via the modulation of TRPV1 function [24]. To further determine the ligand role of osthole on TRPV1, we investigated the interaction between osthole and TRPV1 by molecular docking *in silico* (Figure 4). As shown in Figures 4(a) and 4(b), osthole interacted with TRPV1. The dominant conformation of osthole binding to TRPV1 is located in the hydrophobic pocket of TRPV1. In addition, the binding pattern analysis showed that osthole links with TRPV1 between the S4 and S4-S5 linkers in the binding pocket. Furthermore, osthole formed a hydrophobic interaction with the amino acid residues ALA566, VAL567, and GLN700 (as shown in Figures 4(d) and 4(e)). Osthole formed a strong hydrogen bond interaction with the hydroxyl of ARG557 (1.8–2.0 Å), which is an important residue for opening the TRPV1 channel. The binding energy of osthole was −7.97 kcal/mol, which was slightly higher than that of TRPV1 agonist resiniferatoxin (−11.70 kcal/mol). ARG557 also formed a hydrogen bond with GLU570. The S4-S5 linker was pulled away from the central axis of the TRPV1 ion channel by the hydrogen bond of osthole with ARG557 and the hydrogen bond of ARG557 with GLU570. These results indicate that osthole may slightly open TRPV1.

### 3.3. Osthole-Activated TRPV1 on DRG Neurons

To reveal the direct action of osthole on DRG neurons, we tested the effects of the selective antagonist AMG9810 on TRPV1 on osthole-induced calcium influx. The results demonstrated that AMG9810 (1 *μ*M) blocked the effect of osthole (30 *μ*M) on DRG neurons (Figure 5). As shown in Figures 5(a)–5(c), osthole-induced calcium influx was obvious. However, pretreatment with AMG9810 significantly attenuated the fluorescence intensity induced by second-osthole application compared with first-osthole application (0.10 ± 0.04 (*n* = 146) vs. 0.45 ± 0.06 (*n* = 262), total cells = 1654, ^*∗∗*^*P* < 0.01, *t*-test, *n* = 3 animals) (Figures 5(a)–5(c)). Furthermore, the percentage of positive DRG neurons that responded to osthole also decreased after pretreatment with AMG9810 (17.36 ± 3.04% vs. 9.49 ± 3.61%, total cells = 1654, ^*∗*^*P* < 0.05, *t*-test, *n* = 3 animals) (Figure 5(d)).

### 3.4. Osthole Desensitized Capsaicin-Induced Calcium Influx

To test whether osthole could desensitize TRPV1, we examined the response of neurons to capsaicin with or without pretreatment with 10 *μ*M or 30 *μ*M osthole (Figure 6). The results showed that a single application of 0.1 *μ*M capsaicin induced robust increase in intracellular calcium, and the fluorescence intensity of the DRG neurons was 0.72 ± 0.04 (26.23% positive cells in total cells, *n* = 3 animals). Although pretreatment with 10 *μ*M osthole did not significantly affect the capsaicin reaction, the fluorescence intensity of the DRG neuron response to capsaicin was 0.69 ± 0.05 (6.36% positive cells in total cells, *n* = 3 animals) (Figure 6(a)). However, pretreatment with 30 *μ*M osthole significantly decreased the capsaicin response to 0.57 ± 0.03 (7.50% positive cells in total cells, *n* = 3 animals, ^*∗*^*P* < 0.05, one-way ANOVA followed by Dunnett's test versus capsaicin treated alone) (Figure 6(b)). In addition, after pretreatment with capsaicin, the DRG neuron response to capsaicin again was reduced (0.26 ± 0.06 vs. 0.72 ± 0.04, *n* = 3 animals, ^*∗∗∗*^*P* < 0.001, one-way ANOVA followed by Dunnett's test versus capsaicin treated alone) (Figure 6(c)). The data showed that osthole might dose-dependently desensitize capsaicin-induced calcium influx, which can activate and subsequently desensitize the TRPV1 channel (Figure 6(d)).

### 3.5. Osthole Reduced Scratching Behavior Induced by Histamine, HTMT, and VUF8430

A previous study reported that histamine induced acute scratching behavior [29]. To confirm the antipruritic effect of osthole on histamine-dependent itch, we examined the effect of osthole (1 *μ*M) on histamine (100 *μ*M), H1 receptor agonist HTMT (0.1 *μ*M), and histamine H4 receptor agonist VUF8430 (100 *μ*M)-induced scratching behavior as previously reported [18, 24]. The results showed that histamine induced obvious scratching behavior. However, after pretreatment with osthole, the scratching bouts induced by histamine (80 ± 16, *n* = 8) were significantly attenuated compared with the control (25 ± 11, *n* = 8, ^*∗*^*P* < 0.05, paired *t*-test) (Figures 7(a) and 7(b)). Similar to histamine, the histamine H1 receptor agonist HTMT-induced scratching behavior and the histamine H4 receptor agonist VUF8430-induced scratching behavior were also inhibited by osthole. The scratching bouts of HTMT (0.1 *μ*M) reduced from 108 ± 17 to 40 ± 7 (*n* = 7, ^*∗*^*P* < 0.05, paired *t*-test) (Figures 7(c) and 7(d)). As shown in Figures 7(e) and 7(f), the scratching bouts of VUF8430 (100 *μ*M) decreased from 144 ± 15 to 87 ± 16 (*n* = 6, ^*∗*^*P* < 0.05, paired *t*-test). The results suggested that osthole inhibited histamine-, HTMT-, and VUF8430-induced obvious scratching behavior. TRPV1 is downstream of the histamine-dependent itch signal transduction pathway, combined with the abovementioned research results, suggesting that the inhibition of osthole on histamine-induced itch may occur through TRPV1.

## 4. Discussion

Itchiness is a common symptom or abnormal sensation in atopic dermatitis, urticaria, and cholestasis, and it is involved in many signaling pathways [30]. These pathways can be subdivided into histamine-dependent such and histamine-independent signaling pathways, such as Mas-related G protein-coupled receptors (Mrgprs) and PAR-2 receptors [31]. TRPV1 is a key downstream ionic channel and a target for the treatment of histamine-dependent diseases [32]. Traditional Chinese medicine or natural herb compounds have been used to treat itch or itchy diseases for a long time [33]. It is valuable to identify active ingredients in traditional Chinese medicine for the treatment of pruritus diseases. This study aimed to investigate the antipruritic molecular mechanisms of osthole, the active component of *C. monnieri*, by active TRPV1.

In this study, it is shown that osthole could repeatedly activate the same DRG neurons (Figure 2), although the neurons were weakly desensitized using osthole for the third time. Furthermore, neurons activated by osthole were almost a subpopulation of small-sized isolated DRG neurons in a dose-dependent manner (Figure 3). In our previous study, we demonstrated that osthole attenuated the scratching behavior induced by histamine via the modulation of the TRPV1 channel [24]. These results suggest that TRPV1 may be an important molecule channel for osthole to treat pruritic diseases.

Previous research has reported that the function of TRPV1 agonists seems to be mainly affected by the presence of residues Tyr511, Ser512, Leu515, Phe543, Met547, Thr550, Lys571, Arg 557, and Glu570 in a homologous model [34–36]. Using molecular docking, we found the osthole hydroxyl on Arg557, which is in accordance with a previous study (Figure 4). The binding pocket of TRPV1 comprises three parts. Several hydrophobic residues, including Leu518, Leu547, Phe554, Leu663, and Leu670 formed the upper part of the binding pocket; Tyr511, Met514, and Thr550 formed the middle part; and two charged residues, Glu570 and Arg557, formed the bottom part [36]. Osthole interacting with the hydroxyl hydrophobic residue Arg557 in the bottom part of the binding pocket may open the channel. However, Wang et al. found that evodiamine as a TRPV1 agonist interacted with the binding pocket formed by Ser510, Tyr511, Leu515, Tyr555, Met568, Ile569, Glu570, and Lys571 [37]. In summary, osthole can activate TRPV1 by forming a hydrogen bond interaction with hydrophobic residues.

In the calcium imaging assay, osthole-induced intracellular calcium increase and the percentage of activated neurons were inhibited by the TRPV1 antagonist AMG9810 (Figure 5). It has been suggested that osthole is an agonist of TRPV1. However, the osthole-induced intracellular calcium influx cannot be completely blocked by AMG9810. This may be because osthole activates the other TRP channels. In other studies, osthole inhibited atopic dermatitis chronic itch by directly downregulating TSLP production from keratinocytes or activating warm-temperature Ca^2+^-permeable TRPV3 channels [19, 38]. In addition, the inhibition of TRPV3 by osthole significantly attenuated the scratching behavior induced by either acetone-ether-water (AEW) or histamine [18]. This indicates that TRP channels play an important role in the pharmacological functions of osthole.

Pharmacological desensitization of receptors is essential for reducing neuronal activity. Low-dose capsaicin topical patches have been widely used in treating pain and pruritus diseases through TRPV1 desensitization in clinical settings [8, 9, 11, 12, 39]. The repeated application of the TRPV1 agonist capsaicin or natural compounds such as evodiamine from *Evodia rutaecarpa* Bentham [40], imperatorin from *Angelica dahurica* root [41], and camphor from *Cinnamomum camphora* [42] to DRG neurons can induce desensitization responses.

In this study, the robust calcium influx induced by capsaicin was significantly different after treatment with or without osthole (Figure 6). The abovementioned results showed that the osthole is an agonist of TRPV1 through interaction with the hydroxyl hydrophobic residue Arg557 in the bottom part of the binding pocket, which the antagonist TRPV1 (AMG9810) can also inhibit. Interestingly, calcium influx was induced by capsaicin-desensitized pretreatment with osthole or capsaicin (Figure 6). However, the desensitization effect of osthole was weaker than that of capsaicin (Figure 6). This proved that osthole, an agonist of TRPV1, can exert its pharmacological action by activating and subsequently desensitizing TRPV1. TRPV1 is one of the main targets for treating histamine-dependent itch [1], and drugs that can desensitize TRPV1 may have an inhibitory effect on histamine-dependent itch [40, 41]. The behavior results shown in Figure 7 are consistent with this theory. Scratching behavior induced by histamine and histamine receptor agonists was inhibited by osthole (Figure 7). In our previous study, osthole also inhibited the increase in intracellular calcium caused by histamine and histamine receptor agonists [24]. Combining all the results mentioned above, we speculate that osthole inhibits histamine-dependent itch in which TRPV1 may play a role.

## 5. Conclusions

In summary, the results demonstrated that osthole could activate DRG neurons, and the molecular docking results show that osthole can be coupled to TRPV1 with the hydrophobic residue Arg557 as an agonist. Indeed, the neurons activated by osthole were inhibited by AMG9810, and osthole could desensitize TRPV1. Furthermore, osthole inhibited the histamine-dependent scratching behavior.

## Figures and Tables

**Figure 1:** Chemical structure of osthole. (a) Two-dimensional structure of osthole. (b) Three-dimensional structure of osthole is displayed by the stick model.

**Figure 2:** Osthole increased intracellular calcium in DRG neurons. (a) Representative fluorescence images of osthole-induced changes in the intracellular calcium concentration. control (A) and osthole (B) (scale bar: 20 *μ*m). (b) The representative trace showed that osthole repeatedly induced calcium influx in the same DRG neuron. (c) Fluorescence intensity of osthole induced is 0.34 ± 0.03 (first treated), 0.22 ± 0.05 (second treated), and 0.15 ± 0.05 (third treated) (cells = 114 (positive)/1202 (total), *n* = 3 animals). The mean fluorescence intensity was desensitization by the third application of osthole in the same neurons (^*∗∗*^*P* < 0.01, one-way ANOVA followed by Dunnett's test versus Ost 1st). Ost, osthole.

**Figure 3:** Osthole activated DRG neurons in dose-dependent manner. (a) Representative fluorescence traces of 10 *μ*M osthole-induced changes in DRG neurons. (b) Representative traces of DRG neurons responded to 30 *μ*M osthole. (c) Representative traces of DRG neurons responded to 100 *μ*M osthole. (d) The mean fluorescence intensity of osthole at different doses induced significant intracellular calcium increase. Fluorescence intensity of osthole at 10 *μ*M is 0.29 ± 0.03 (cells = 161 (positive)/1785 (total), *n* = 3 animals), at 30 *μ*M is 0.43 ± 0.04 (cells = 389 (positive)/2169 (total), *n* = 3 animals), and at 100 *μ*M is 0.62 ± 0.09 (cells = 451 (positive)/1540 (total), *n* = 3 animals) (^*∗*^*P* < 0.05, *t*-test, 10 *μ*M osthole versus 30 *μ*M osthole; 30 *μ*M osthole versus 100 *μ*M osthole).

**Figure 4:** Molecular docking of osthole combined with TRPV1. (a) The docking site based on the structure of TRPV1 protein active site. The green band represents TRPV1, and the yellow stick means the key residue of the active site. The overlapping display of 48 docking conformations of osthole on the activated site of TRPV1 is shown. The blue represents the docking conformation. (b) Combination model of osthole with TRPV1. Left: the surface of TRPV1, and the yellow stick represents osthole. Right: the gray band represents TRPV1, and the yellow stick represents osthole. (c–e) Chemical bond of osthole combined with TRPV1. (c) The hydrophobic interaction of osthole and TRPV1. Orange represents highly hydrophobic area, blue represents highly hydrophilic area, and the yellow ball-stick represents osthole. (d) The two-dimension schematic representation of the interaction between osthole and residues of TRPV1 protein's activated site. (e) The three-dimensional interaction structure of osthole and TRPV1.

**Figure 5:** Osthole induced calcium influx through TRPV1 in DRG neurons. (a) Representative images in cultured DRG neurons at normal (aA) and after treatment with osthole (30 *μ*M) (aB), pretreatment with AMG9810 (1 *μ*M) (AMG9810 + osthole) (aC). Kcl (aD) was used as the positive control (scale bar: 20 *μ*m). (b) Representative traces showed the neurons activated by osthole were inhibited by pretreatment of TRPV1 antagonist AMG9810. (c) The mean fluorescence intensity of osthole positive neurons were restrained by pretreatment of AMG9810 (0.45 ± 0.06 (*n* = 262) vs 0.10 ± 0.04 (*n* = 146), total cells = 1654, ^∗∗^*P* < 0.01, *n* = 3 animals). (d) The percentage of osthole positive neurons was inhibited by pretreatment of AMG9810 (17.36 ± 3.04% vs 9.49 ± 3.61%, ^∗^*P* < 0.05, total cells = 1654, *n* = 3 animals).

**Figure 6:** Osthole desensitized capsaicin-induced calcium influx. (a, b) Representative traces showed the effect of pretreatment with 10 *μ*M and 30 *μ*M osthole on capsaicin-induced calcium influx. (c) Representative traces showed the effect of pretreatment capsaicin on secondary capsaicin-induced calcium influx. (d) The mean amplitudes of capsaicin-induced calcium influx were significantly different with pretreatment of osthole or capsaicin. Fluorescence intensity of capsaicin treated alone is 0.72 ± 0.04 and treated secondly is 0.26 ± 0.06 (cells = 161 (positive)/1785 (total), *n* = 3 animals). Fluorescence intensities of capsaicin after treatment with 10 *μ*M and 30 *μ*M osthole are 0.69 ± 0.05 (cells = 106 (positive)/1650 (total), *n* = 3 animals) and 0.57 ± 0.03 (cells = 102 (positive)/1360 (total), *n* = 3 animals). Cap, capsaicin (^*∗*^*P* < 0.05, ^*∗∗∗*^*P* < 0.001, one-way ANOVA followed by Dunnett's test versus capsaicin treated alone).

**Figure 7:** Osthole attenuated the scratching behavior induced by histamine, HTMT, and VUF8430. Histamine, HTMT, and VUF8430 induced scratch behavioral with or without pretreatment with osthole. Time course of itch-related behaviors during 30 minutes (a, c, e) and total scratch bouts (b, d, f) is shown. Osthole significantly inhibited the scratching behavior induced by histamine in mice in 30 minutes (*n* = 8) (a, b). Similar to histamine, HTMT-induced obvious scratching behaviors were significantly attenuated by osthole (*n* = 7) (c, d). Osthole also inhibited the VUF8430-induced scratching behavior in mice (*n* = 6) (e, f) (^*∗*^*P* < 0.05, pair *t*-test).

## Data Availability

The data used to support the findings of this study are included within the article.
